# Human and Environmental Dangers Posed by Ongoing Global Tropospheric Aerosolized Particulates for Weather Modification

**DOI:** 10.3389/fpubh.2016.00139

**Published:** 2016-06-30

**Authors:** J. Marvin Herndon

**Affiliations:** ^1^Transdyne Corporation, San Diego, CA, USA

**Keywords:** geoengineering, coal fly ash, aerosol particulates, autism spectrum disorder (ASD), Alzheimer’s disease, Parkinson’s disease, neurological disorders, chemically mobile aluminum

## Abstract

**Background:**

U.S. military perception of nuclear warfare led to countless unethical nuclear experiments performed on unsuspecting individuals without their informed consent. As evidenced here, subsequent perception of weather warfare has led to exposing millions of unsuspecting individuals to toxic coal fly ash with no public disclosure, no informed consent, and no health warnings.

**Methods:**

Three methods were used: (1) comparison of eight elements analyzed in rainwater samples, thought to have leached from aerosolized coal fly ash, with corresponding coal fly ash laboratory leachate; (2) comparison of 14 elements analyzed in air filter dust with corresponding elements in coal fly ash; and (3) comparison of 23 elements analyzed in fibrous mesh found after snow melted with corresponding elements in coal fly ash.

**Results:**

The rainwater element ratios show that the aerial particulate matter has essentially the same water-leach characteristics as coal fly ash. The air filter dust element ratios occur in the same range of compositions as coal fly ash, as do element ratios in fibrous mesh found on grass after snow melted. The fibrous mesh provides an inferred direct connection with the aerosolizing jet aircraft *via* coal fly ash association with the jet combustion environment.

**Conclusion:**

Strong evidence for the correctness of the hypothesis: coal fly ash is likely the aerosolized particulate emplaced in the troposphere for geoengineering, weather modification, and/or climate alteration purposes. The documented public health associations for ≤2.5 μm particulate pollution are also applicable to aerosolized coal fly ash. The ability of coal fly ash to release aluminum in a chemically mobile form upon exposure to water or body moisture has potentially grave human and environmental consequences over a broad spectrum, including implications for neurological diseases and biota debilitation. The ability of coal fly ash to release heavy metals and radioactive elements upon exposure to body moisture has potentially grave human health implications including cancer, cardiovascular disease, diabetes, respiratory diseases, reduced male fertility, and stroke. The fibrous mesh data admit the possibility of environmentally disastrous formation of methylmercury and ozone-depleting chlorinated-fluorinated hydrocarbons in jet exhaust. Geophysical implications include atmospheric warming and rainfall retardation.

## Introduction

In a civilized, humanitarian society, public health responsibilities include revealing threats that arise from both biological and anthropogenic causes. Global-scale naturally caused public health threats have long existed, are generally well known, and have been the subject of scholarly research. Far-reaching human-caused threats to public health, on the other hand, have mainly occurred since World War II and are typically the result of deliberate military activities conducted secretly. Public disclosure of military-originated public health dangers by scientists has galvanized public outrage against such activities in the past. The Manhattan Project gave rise to the nuclear arms race. Unethical nuclear experiments were performed involving unsuspecting individuals, sometimes numbering in the thousands, without informed consent. For example, pregnant women, told they were receiving vitamins, were instead given radioactive iron; newborn infants were injected with radioactive iodine-131 (1–4). Atmospheric detonations of nuclear devices were generally undertaken without regard for the health of unsuspecting residents downwind (5). Atmospheric nuclear testing in the United States ended as a consequence of the public outcry over civilian public health disclosure of the risks associated with strontium-90 uptake by children (6).

Modern commercial weather modification technology began with the 1946 discovery that clouds, seeded with silver iodide or dry ice, could be caused in many instances to yield rain or snow (7). That weather modification method is widely used for agricultural and other commercial purposes. Ski resorts frequently use it to increase the likelihood of snow. Insurance companies use it to cut their risks when guaranteeing certain weather conditions for commercial projects or to minimize potential losses caused by hail storms.

The military has long dreamed of controlling the weather for strategic purposes (8). The early military applications of weather modification were aimed at deliberately causing rainfall at a specific time and place by cloud seeding with substances such as silver iodide or dry ice. Reportedly, the U.S. seeded clouds to squeeze rain out before they reached Cuba in order to ruin the Cuban sugar cane harvest (9). From 1967 to 1972, Operation Popeye involved cloud seeding with the intention of extending the monsoon season over the Ho Chi Minh Trail to impede transport of troops and supplies during the Vietnam War (8, 10). The success of these weather modification activities provided impetus for the subsequent government/military technological interests, expressed in a 1978 U.S. Senate document (11) and described in the 1996 U.S. Air Force document: “Weather as a Force Multiplier: Owning the Weather in 2025 (12).”

After the Vietnam War, military weather modification became a secret global-scale activity buttressed by a campaign of disinformation. Like its nuclear-warfare predecessor, weather modification or geoengineering continued to be covertly developed and practiced, especially over the past two decades (13). That geoengineering activity poses global-*scale* public-health dangers due to the nature of the principal substance being sprayed into the lower atmosphere, troposphere (14), where it mixes with the air we all breathe (15) (Figure 1). The government not only hides the known (and unknown) health risks but also misleads the public about its geoengineering program and the nature of the aerosol substances it employs.^1^

**Figure 1:** **Schematic representation of atmosphere layers at mid-latitudes showing typical regions of cloud formations and passenger jet traffic**.

Nevertheless, through application of forensic-science methodologies and with sound observations and scientific reasoning, crucial aspects of the covert tropospheric spraying activities can be discerned. For humanity’s sake, the public health and environmental implications of the current on-going, global-scale, covert tropospheric spraying are herewith disclosed for public discussion, research, and verification.

A profound dichotomy exists between the technology, practice, terminology, and public disclosure of geoengineering so that public discussion of its implications for public health is minimized. The academic community describes geoengineering as a possible *future* intervention in the upper atmosphere (stratosphere) to counteract anthropogenic global warming. The stratosphere is the region where volcanic eruption gases have been observed to cause global cooling. There is relatively little convection in the stratosphere so volcanic ejecta can stay suspended in the stratosphere for a year or more (16). Academic scientists postulate future geoengineering in which substances such as sulfuric acid or titanium dioxide are sprayed into the stratosphere in order to block a portion of incident sunlight (17). Various methods have been proposed for emplacing geoengineering substances into the stratosphere including shooting the substances from guns or releasing them from balloons or high-altitude jets (18). The stratosphere is the region harboring the ozone-layer that protects us from the ultraviolet component of sunlight (19). Within the academic perception of hypothetical geoengineering, public health concerns arising from geoengineering are also hypothetical, something that may become important in the future if and when stratospheric geoengineering is put into practice.

In contrast to the presumption of academic geoengineers, covert government/military geoengineering activity has occurred over the past 70 years and has intensified since the end of the Cold War and the discovery of global warming as a national security issue (20). Currently, geoengineering is taking place in the troposphere (lower atmosphere) over a large number of countries, including the United States, Canada, the European Union countries, England, Australia, and New Zealand (14). The academic community has been hesitant to publically acknowledge military geoengineering activity even though there is abundant observational evidence for its existence (8, 14). Since the mid-1990s, there have been numerous observations of aerial spraying of particulate matter in the troposphere. Figure 2 shows some recent examples of the particulate trails; however, this is a minuscule sampling. There are numerous websites devoted to exposing aerial spraying to the uninformed public.^2^^–^^14^

**Figure 2:** **Images of deliberately produced particulate pollution trails**. Photographs by Patrick Roddie, with permission.

The physical basis for particulate aerial spraying is to control weather and climate by inhibiting rain. The idea behind cloud seeding is *to aid* the nucleation of rain, ice, or snow whereas the idea behind aerosolized particulate spraying to inhibit rainfall is *to interfere* with the nucleation process. The methodology is known from pollution studies (21) and is described by NASA^15^: “Normal rainfall droplet creation involves water vapor condensing on particles in clouds. The droplets eventually coalesce together to form drops large enough to fall to Earth. However, as more and more pollution particles (aerosols) enter a rain cloud, the same amount of water becomes spread out. These smaller water droplets float with the air and are prevented from coalescing and growing large enough for a raindrop. Thus, the cloud yields less rainfall over the course of its lifetime compared to a clean (non-polluted) cloud of the same size.”

The government/military solution to inhibit the fall of rain is to deliberately add an aerosolized pollutant to the region where clouds form to interfere with raindrop nucleation. The intentional addition of particulate pollution not only inhibits the fall of rain but also warms the atmosphere (by absorbing solar energy) and limits loss of heat radiated by Earth. Consequently, the particulate pollution creates an artificial increase in air pressure, which can block the movement of an oncoming weather front thus further keeping the sprayed area from experiencing rainfall (22, 23). Subsequent settling of the pollutant matter on ice sheets may serve as solar heat collectors and aid in melting the ice (24). The harm to citizens, plants, and other biota comes not only from decreased precipitation but also from the toxic content of the pollutant substance widely utilized to retard the fall of rain (25).

The composition of the aerosolized particulate matter, often referred to as “chemtrails,” to distinguish them from contrails, has been a closely guarded secret, and accompanied by a disinformation campaign. For example, in 2005, the U.S. Air Force distributed a document entitled “Contrails Facts”, which asserted in part: “The ‘Chemtrail’ hoax has been investigated and refuted by many established and accredited universities, scientific organizations, and major media publications. There is no such thing as a ‘Chemtrail.’ Contrails are safe and are a natural phenomenon. They pose no health hazard of any kind.”

But as Abraham Lincoln famously said, “You can fool all the people some of the time, and some of the people all the time, but you cannot fool all the people all the time.” On February 11, 2016, a bill was introduced into the General Assembly of the State of Rhode Island (USA) that would demand public disclosure and health and safety evaluations of any geoengineering activities (26). On March 11, 2016, a mass-tort environmental proposed Class Proceeding (“Proceeding”) was brought in the Federal Court of Canada on behalf of all affected Canadians in respect of Aerial Discharges performed directly or indirectly by Her Majesty the Queen and/or her instrumentalities, in Canadian air space, and which Aerial Discharges are alleged to compromise cognitive function, contribute to other neurological disorders, damage property and the environment, among many other heads of damage (27).

The aerial graffiti superficially resembles contrails, which are ice crystals formed from aircraft exhaust, but there are profound differences. Contrails only form in very humid environments, with temperatures low enough for the saturation vapor pressure with respect to ice, and with sufficient moisture content in the exhaust gases. Moreover, the ice crystals that form contrails sublimate, disappearing by evaporation to form invisible gas on a time scale ranging from seconds to minutes (typical) to a few hours (extremes of cold and humidity) (28, 29).

The author has lived in San Diego, California (USA) for more than 40 years and as a trained scientist keenly observes the sky. For many years before the near-daily particulate spraying, the sky overhead was a rich azure blue color, frequently without clouds. In the warm dry air above San Diego, jet contrails are a rare sight that disappear in a matter of seconds to minutes, becoming invisible gas. Figure 3 shows six images of the San Diego sky that not only illustrate the nature of the now-pervasive particulate spraying but clearly provide the basis to refute the Air Force’s published statement. Videos of aircraft spraying particulate matter into the San Diego sky are referenced here.^16^^–^^20^

**Figure 3:** **Photographs of the sky above San Diego, California (USA) taken in 2014–2015**. Top left: note the mainly blue sky, with a just small amount of white haze. Top right: spray stopped in mid-flight, which is uncharacteristic of jet contrails. Middle left: heavy spraying produced artificial overcast of an otherwise cloudless blue sky. Middle right: heavy spraying changed the blue sky to overcast with a brownish hue. Bottom left: numerous particulate trails unlike paths of normal air traffic. Bottom right: note the white haze caused by micron and sub-micron size particulates, which is uncharacteristic of jet contrails, ice crystals that rapidly disappear by evaporation. The blue stripe copied from the top left image shows the contrast. Before the heavy aerial spraying began, San Diego skies were usually the color of the blue stripe and often without cloud cover. The warm dry climate above San Diego prevents the formation of persistent jet contrails, which are ice crystals.

All of the photographs that comprise Figure 3 were taken on days with no natural clouds in the San Diego sky. The top left image of Figure 3 shows a section of rich azure blue San Diego sky with little evidence of particulate spraying. The top right image shows two trails crossing in the same region of sky, hence in similar environments, but one abruptly ceases, while the other does not. That is not the behavior of contrails, which would have behaved similarly, but rather the operation of particulate sprays where one was shut off or ran out of feedstock. Note the wispy cirrus-like “clouds” in the background. Soon after the particulate trail is laid, it begins to diffuse initially forming cirrus-like artificial clouds, which then further diffuses to form a white haze in the sky. The middle left photograph was taken after heavy spraying throughout the day produced an artificial overcast. The middle right photograph shows even heavier spraying that produced artificial overcast with a brownish hue. The lower left shows multiple particulate trails over a recognizable location in San Diego that is uncharacteristic of normal jet traffic patterns. The lower right image shows the typical white haze produced by the particulate sprays. The blue strip at the top of the image, from the top left photo, shows for comparison natural un-polluted San Diego sky. Jet contrails do not produce white haze in San Diego skies.

Even without knowing the identity of the specific particulate matter being sprayed into the air we breathe, we may infer the potential of major adverse health risks from aerosolized particulates because they are similar in size to air pollution particles the health effects of which have been extensively studied (30). For aerosolized particulates to remain suspended for some period of time before settling, the particles must be micron (μm) or submicron in size (31). As known from epidemiological studies, pollution particles with similar diameters, ≤2.5 μm, referred to as PM_2.5_, have been found to be associated with increased hospital admissions (32), morbidity and premature mortality (33–35), risk for cardiovascular disease (36) and lung cancer (37), lung inflammation and diabetes (38), risk for stroke (39), Alzheimer’s disease (40, 41), onset of asthma (42), renal function in older men (43), low birth weight (44), and reduced male fertility (45).

The author published the first paper in the peer-reviewed scientific literature that provided initial evidence that the main substance being aerosolized for military tropospheric geoengineering is coal combustion fly ash (14). The purpose of the present paper is to provide considerably more scientific evidence that the aerosolized particulate matter is coal fly ash, and offer considerably greater insight to the public health risks and environment impact of this multi-component aerial pollutant.

Industrial coal burning produces four kinds of waste products: (1) heavy bottom ash that settles out; (2) micron and sub-micron size particles, called coal fly ash that would go up the smokestack unless electrostatically captured and stored as is presently mandated in Western nations (46, 47); (3) boiler slag; and (4) flue gas desulfurization product (gypsum). Of these, coal fly ash is by far the most toxic substance. When coal formed it trapped a great variety of toxic elements. Much of coal’s toxic component is released upon burning and incorporated in coal fly ash, making coal fly ash a toxic nightmare capable of releasing many toxins upon exposure to water (48). These toxins include aluminum in a chemically mobile form, which is implicated in human neurological diseases (49–51) and biota distress (52, 53). “Forest die-offs and reduced survivorship or impaired reproduction of aquatic invertebrates, fish, and amphibians have been directly connected to Al toxicity. Indirect effects on birds and mammals also have been identified (54).”

Coal fly ash is a major industrial waste stream for Western nations’ coal-fired electric utilities. Notably, coal fly ash has the appropriate grain-size distribution for aerosolized tropospheric spraying or else it is relatively simple to further separate an extra-fine component using cyclone classifiers (separators). Huge quantities of coal fly ash are readily available worldwide at extremely low cost. Moreover, electrostatic trapping and processing facilities, as well as transport infrastructure, are in place and generally out of public view. The author submits the following hypothesis: coal fly ash is likely the principal aerosolized particulate sprayed in the troposphere by jets for geoengineering, weather modification, and/or climate alteration purposes.

The objectives of the author’s research are fourfold: (1) to provide further scientific evidence as to the correctness of the hypothesis that coal fly ash is likely the aerosolized particulate sprayed in the troposphere for geoengineering, weather-modification, and/or climate-modification purposes; (2) to reveal some of the adverse human public health consequences and the antagonistic consequences on Earth’s environment and biota; (3) to provide evidence that, in addition to being directly discharged into the atmosphere, coal fly ash may be exposed to jet fuel combustion environment prior to being dispersed; and, (4) to suggest that ozone-destructive chlorinated-fluorinated hydrocarbons and toxic methylmercury (CH_3_Hg) may be produced when coal fly ash is exposed to the jet fuel combustion environment.

## Materials and Methods

The methodology is threefold: (1) compare the element ratios analyzed in rainwater with corresponding element ratios analyzed in the leachate of coal fly ash laboratory leach experiments (48, 55); (2) compare the element ratios analyzed in dust collected outdoors by high-efficiency particulate arresting (HEPA) air filters with corresponding element ratios analyzed in samples of coal fly ash; and (3) compare the element ratios analyzed in fibrous matter collected on grass after snow melted away with corresponding element ratios analyzed in samples of coal fly ash.

Since at least 2002, individuals have collected post-spraying rainwater for chemical analysis (see footnote text 2–5). Usually only aluminum analyses were requested, but sometimes also barium, and more rarely strontium were also included in the analysis request. In 2015, the author published the first paper showing that for those three-element rainwater analyses, the ratios Al/Ba and Sr/Ba compare favorably with similar ratios from analyses of the leachate from laboratory coal fly ash leaching experiments (14). Here, the author compares three separate San Diego (USA) post-spraying rainwater analyses for Al/Ba, Sr/Ba, Fe/Ba, Ca/Br, S/Br, Mg/Br, and B/Br with corresponding coal fly ash leachate ratios.

Since at least 2008, a few individuals have trapped air-borne particles on HEPA filters and had the dust analyzed. Here, the author compares the analytical results from four samples, expressed as element ratios relative to barium, with corresponding ratios from analyses of coal fly ash.

Occasionally fibers, sometimes referred to as “spider webs,” are observed descending from above, swept along by the wind, trapped on vegetation, and on the ground;^21^^–^^24^ some observers have speculated that these originated from aerial spraying. Recently, such fibers were found on grass as snow was melting away and were collected and analyzed. Here, the author compares those analytical results, expressed as ratios relative to barium, with corresponding ratios from analyses of coal fly ash.

## Results

Coal fly ash is trapped and confined in Western countries because it contains numerous toxic elements including aluminum, arsenic, barium, cadmium, chromium, lead, mercury, selenium, thorium, and uranium among others. These elements are readily released by contact with water. Moreno et al. (48) conducted leaching experiments on 23 different coal fly ash samples from European sources (Spain, The Netherlands, Italy, and Greece), which they analyzed for 33 elements. They leached 100 g of each sample in 1 liter of distilled water in a 2-liter bottle for 24 h. They then analyzed the filtered leachate solution of each for 38 elements. No reason was given for the greater number of leachate analyses. These data provide the primary standard for comparison of the analytical results for rainwater, HEPA filter dust, and fibrous matter reported here. An additional comparison is made of the range of compositions and range of leachate values of 12 American coal fly ash samples, ten of which come from the Illinois Basin (55).

### Rainwater

Before the near-daily aerial spraying in San Diego, California (USA), where the author has resided for more than 40 years, on many days of the year the skies were blue, cloudless and without the white haze that is the consequence of the aerial spraying; now, the visual effects of the spraying are clearly evident (Figure 3). The author collected San Diego rainwater samples in February, May, and December 2015 for analysis. San Diego is ideal for rainwater sample collection as there are no coal-burning facilities nearby or in the path of prevailing winds and there are no heavy industries to cause air borne pollution in San Diego. The residence-time for smokestack particulates in the boundary layer, a few days at most, is too short for coal fly ash to arrive from China *via* low-level transport, which takes longer than 10 days (56). Further, the observed aerial particulate density, at times sufficient to cause artificial overcast (Figure 3), is related to observed aircraft spraying activities, and is not present in the absence of aerial activity.

The rainwater samples were sent to two commercial state-of-California certified laboratories, Babcock Laboratories, Inc., and Basic Laboratory. Their analytical results, by inductively coupled plasma mass spectrometry, were consistent to within 2–10%. Figure 4 shows the San Diego rainwater analytical element ratios for comparison with corresponding ratios of the average values and ranges of the Moreno et al. (48) laboratory leachate results for 23 European coal fly ash samples and the range of American coal fly ash leachate data of Suloway et al. (55). The European coal fly ash samples were leached using distilled water (pH = 7.00). After leaching for 24 h the pH of the 23 laboratory leachates ranged from 6.40 to 12.54. Comparable data are not available for the American leach experiments as the pH was constantly adjusted during the experiment to maintain a value of 5.00. Figure 4 also includes for comparison the analytical rainwater results from Internet sources (see footnote text 2–5) published by the author (14, 57). Plotted data are shown in Tables 1–3.

**Figure 4:** **Analyzed element ratios in San Diego rainwater samples taken in February, May, and December of 2015 shown for comparison with the range of corresponding element ratios and average values from laboratory coal fly ash leachate of 23 European (48) and 12 American coal fly ash samples (55)**. Previously published (14) rainwater Al/Ba and Sr/Ba ratios from Internet postings are shown for comparison.

**Table 1:** **Analytical ICP-MS data for San Diego rainwater samples**.

		February 2015 μg/liter	May 2015 μg/liter	December 2015 μg/liter
Aluminum	Al	41	26.3	88.9
Barium	Ba	5.3	3.2	10.1
Boron	B	18.2	9.1	48.2
Calcium	Ca	1600	1200	3300
Iron	Fe	38	14	78
Magnesium	Mg	800	800	2700
Strontium	Sr	7.2	6.3	19
Sulfur	S	540	815	1860

*The differences between samples primarily reflect various amounts of dilution*.

**Table 2:** **Tabulation of Internet-posted ICP-MS analytical data plotted in Figure 4**.

Aluminum μg/liter	Barium μg/liter	Strontium μg/liter	Al/Ba Ratio	Sr/Ba Ratio
14	13	110	1.08	8.46
68	33	190	2.06	5.76
28	5	8.9	5.6	1.78
280	32	54	8.75	1.69
7.3	0.84	0.89	8.69	1.06
400	39.1	30.1	10.2	0.77
620	95	59	6.53	0.62
44	5.8	3.4	7.59	0.59
368	6	3	61.3	0.5
2190	43		50.9	
1010	8		126	
700	23.9		29.3	
650	10		65	
219	257		0.85	
188	7		26.9	
140	47		2.98	
118	3.9		30.3	
88.7	4.1		21.6	
66.9	2.1		31.9	
60	10		6	
33.2	3.9		8.5	
27.2	1.6		17	
58	2.5		23.2	
20.2	4.7		4.3	
8	9		0.9	
7.8	0.93		8.4	

*Data sources (see footnote text 2–5)*.

**Table 3:** **Analytical ICP-MS data for HEPA filter dust and fibers**.

		Los Angeles μg/filter	Montebello μg/filter	Pheonix 2009 μg/g	Pheonix 2008 μg/g	Fibers μg/g
Aluminum	Al	5030	1200	39000	12800	4600
Antimony	Sb	29.9	4.19	26		
Arsenic	As	4.66	1.07	48		40
Barium	Ba	344	57.9	2100	556	100
Beryllium	Be					0.2
Cadmium	Cd	1.69		1.7	1.25	0.35
Calcium	Ca			30600	40400	7400
Chromium	Cr	28.4	4.2	48	28.2	56
Cobalt	Co	5.46	0.696	14		3.2
Copper	Cu	387	42.1	172	197	150
Iron	Fe			17300	16800	10000
Lead	Pb	105	26	56	50.5	15
Lithium	Li			15		
Magnesium	Mg			9900	10600	3000
Manganese	Mn			487	562	370
Molybdenum	Mo	12.4	1.5	4		1.7
Nickel	Ni	17.6	6.01	34	33.8	13
Potassium	K			2700	7930	4700
Selenium	Se	3.8	1.08			
Silicon	Si				1020	940
Sodium	Na			1200	6370	410
Strontium	Sr			178	245	47
Titanium	Ti			1900		280
Vanadium	V	29	5.43	46	31.2	14
Zinc	Zn	727	119	1100	593	170

*Sample weights unspecified in reports*.

Ranges of variations are observed in the compositions of coal fly ash (48, 55). These variations arise not only from differences in coal type, in chemical compositions and mineral constituents of the coal from the various locations, but also arise from fly ash characteristics and from boiler configurations and prevailing physical conditions during the burning process. Despite those variable factors, there is nevertheless an overall compositional consistency. Not surprisingly, overall compositional consistency appears to be the case as well for leachate compositions leached from coal fly ash samples from different locations. Note in Figure 4 that the Internet-posted rainwater Al/Ba ratios (14), determined on samples from the United States, France, and New Zealand, are quite similar to the San Diego rainwater Al/Ba ratio and span a range less than the corresponding leachate range of the 23 European coal fly ash samples. A similar observation may be made with respect to the published rainwater Sr/Ba ratios. Indeed, each of the seven San Diego rainwater ratios of the three data sets is remarkably similar to the corresponding European leachate average and range. Rainwater samples absent aerial spraying would be desirable as blanks, but the near-daily, pervasive spraying makes such samples impossible to obtain.

Do the data shown in Figure 4 prove that the aerosolized substance is indeed coal fly ash? Not necessarily, as incontrovertible proof is difficult to obtain, except in mathematics. But the data of Figure 4 do show that some substance in the atmosphere is capable of being leached by rainwater and that substance has for eight elements similar leach characteristics to coal fly ash.

### HEPA Air Filter Dust

Citizens throughout Western nations, concerned about the particulate spraying they observe in the troposphere, have taken numerous samples other than rainwater. Some instances, such as soil samples, are too complicated to draw meaningful conclusions. In many instances, though, too few elements were ordered in the analyses. Individuals in Los Angeles and Montebello, California (USA) in 2011, and in Phoenix, Arizona (USA) in 2008 and 2009 were exceptions. During times of intense aerial spraying these citizens ran HEPA air filters out doors for 3 months during times of intense aerial spraying to capture air borne dust which they had analyzed for 14 chemical elements by state-certified laboratories. The laboratory results were posted on the Internet, but led to no immediately conclusions other than that a number of toxic elements were evident.

Having had the experience of comparing post-spraying rainwater analyses to laboratory-produced coal fly ash leachate, the author decided to compare the HEPA air filter analyses with corresponding analyses of non-leached coal fly ash samples (48, 55, 57). As in the case of San Diego, there were no coal burning facilities and no polluting heavy industries nearby or in the path of prevailing winds for the Los Angeles, Montebello, and Phoenix areas where sample collections took place. As noted above, the residence-time for smokestack particulates in the boundary layer, a few days at most, is too short for coal fly ash to arrive from China *via* low-level transport, which takes longer than 10 days (56).

Figure 5 shows the comparisons of the four sets of analyses of HEPA air filter dust, normalized to barium, with corresponding ratios of the average and range of European coal fly ash compositions from Moreno et al. (48) and from a suite of 12 investigated by Suloway et al. (55) that includes ten from the Illinois Basin (USA), one from North Dakoda (USA) and one from Minnesota (USA). Even though coal fly ash varies in composition according to location, the data presented in Figure 5 show the great similarity between the four samples of HEPA filter dust and coal fly ash compositional ranges. That great similarity is further evidence in support of the following hypothesis: coal fly ash is likely the principal aerosolized particulate sprayed in the troposphere by jets for geoengineering, weather modification, and/or climate alteration.

**Figure 5:** **Analyzed element ratios of dust collected on four high-efficiency air filters shown for comparison with the range of corresponding element ratios and average values for 23 non-leached European coal fly ash samples (48) and element ratio ranges of 12 U.S. coal fly ash samples (55)**. Also shown, 11 of 22 element ratios of fibrous mesh (Figure 6); remaining 11 element ratios are shown in Figure 7.

It follows logically that if aerosolized coal fly ash is the progenitor of the rainwater content of aluminum, barium, strontium, and other elements by leaching, as evidence suggests (Figure 4), then coal fly ash should be found trapped on HEPA air filters (Figure 5) as the tropospheric air at spray-altitudes mixes with the air we breathe (15).

### Fibers Found after Snow Melted

In the spring of 2015 a citizen in Laona, Wisconsin (USA) noticed that immediately after snow had melted a fibrous, sticky mesh, initially flexible and sticky, covered the underlying grass (Figure 6). Upon drying over a period of 24 h, the white fibrous mesh became brittle; subsequent addition of water decomposed the fibrous mesh into a black gelatinous mass. Samples of the brittle white fibrous mesh were analyzed by inductively coupled plasma mass spectrometry at Northern Lake Services, Inc. in Crandon, Wisconsin. Of the 26 elements detected and measured in the fibrous mesh, 23 had been measured by Moreno et al. (48) in the non-leached coal fly ash European samples. Of the 22 element ratios relative to barium that are common to each data set, 11 are common to element ratios measured in HEPA air filter dust and are shown with those ratios in Figure 5. Considering the compositional variability in coal fly ash from different sources, it is reasonable to conclude that the fibrous mesh ratios are essentially indistinguishable from ratios measured in the HEPA air filter data and in turn are essentially indistinguishable from ratios measured in non-leached coal fly ash. Figure 7 is a comparison of the remaining 11 fibrous mesh ratios with corresponding ratios of the average and range of European coal fly ash compositions from Moreno et al. (48) and American coal fly ash composition ranges published by Suloway et al. (55). The great similarity observed in the data plotted in Figure 7 further reinforces the assertion that the composition of the white fibrous mesh is essentially identical to that of coal fly ash.

**Figure 6:** **Photographs of fibrous mesh observed atop grass just as snow had melted showing its initially “sticky” nature**. Photos by Robert West, with permission.

**Figure 7:** **Remaining 11 of 22 analyzed element ratios of fibrous mesh found after snow had melted (Figure 6) shown for comparison with the range of corresponding element ratios and average values for 23 non-leached European coal fly ash samples (48) and element ratio ranges of 12 U.S. coal fly ash samples (55)**. See Figure 5 for the other 11 of 22 element ratios of fibrous mesh.

Coal fly ash is electrostatically trapped as a powder that ranges in color from tan to dark gray depending on composition, which is consistent with observations of the dust trapped by HEPA air filters, which is further consistent with the hypothesis that coal fly ash is sprayed from jet aircraft. So, how might one account for the strikingly different appearance of the fibrous mesh morphology if indeed it is, as evidence indicates, essentially identical in composition to coal fly ash? For the reasons and observations described in the next section, the author posits potential circumstances in which coal fly ash is sometimes exposed to jet fuel combustion, which usually leads to aerosolized coal fly ash, but occasionally, depending physical variables, leads to the production for fibers instead. Viewed this way, the fibrous mesh provides an inferred direct connection with the aerosolizing jet aircraft and also admits the possibility for further investigation of environmentally disastrous formation of methylmercury (CH_3_Hg) and/or the production of ozone-depleting chlorinated-fluorinated hydrocarbons in the jet exhaust.

## Discussion

The analytical results reported for rainwater (Figure 4), airborne particulates collected on HEPA air filters (Figure 5), and the fibrous mesh (Figures 4 and 6) stand as evidence that coal fly ash is the principal material emplaced in the troposphere for ongoing, covert geoengineering, weather modification, and/or climate alteration. For more precise information, future experiments should sample airborne particulates at the altitude in which they are being dispersed into the atmosphere. Alternatively, the nature of the substances being sprayed into the air people breathe may be sought through the process of judicial discovery in legal proceedings such as recently initiated in Canada (27).

### Biotic and Public Health Consequences of Tropospheric Spraying

The ultra-fine particles of aerosolized coal fly ash do not long remain at the altitudes they are emplaced in the troposphere. The particles mix with and pollute the air people breathe (15) and contaminate the soil with toxic, soluble aluminum. The coal fly ash also causes pH changes in the soil. Aluminum is an abundant element in Earth’s crust, but typically it is tightly bound to oxygen and other elements. Earth’s biota evolved without adapting defense mechanisms for soluble aluminum compounds. Tropospheric aerosolized coal fly ash poses environmental health threats from aluminum similar to those posed by acid rain, but without necessarily requiring an acid environment. The pH of coal fly ash varies and can be acidic or basic depending on its coal source. Eastern USA bituminous coal fly ash, for example, has been found to be acidic with pH in the range of 4.3–4.9 (58), whereas coal fly ash from the Western USA tends to be more basic, with pH in the range 8.16–12.4 according to one study (59). Uncontaminated natural rainwater has an acidic pH of about 5.7 due to interaction with atmospheric CO_2_ (60); however, an acidic pH is not a required to leach toxins from coal fly ash. In the experiments on European coal fly ash samples by Moreno et al. (48), distilled water led to aluminum extraction while other chemicals extracted led to leachate pH values in the range 6.2–12.5.

Before action was taken to prevent acid rain (61), chemically mobile aluminum, which is soluble in water, was released into the environment from geological sources, such as mine tailings, and caused serious adverse effects on forests. Forest die-backs in North America were attributed to aluminum toxicity. These blighted forests included balsam fir, Fraser fir, loblolly pine, red spruce, slash pine, and sugar maples (54). Whereas reductions in NO*_x_* and SO_2_ emissions have seriously reduced the acid rain threat, there is a global decline in large old trees (62) and particularly in the Western USA (63). The biochemical–geochemical cycling of aluminum is complex. Its dissolved form is most readily assimilated by living organisms. Once in solution, aluminum may combine with several organic complexes, especially oxalic, humic, and fulvic acids. The metal may also combine with inorganic anions including sulfates, fluorides, phosphates, bicarbonates, or hydroxides, depending on their relative concentrations. Biological activity and toxicity vary with composition and pH. Generally, sulfates are less toxic than hydroxide or organically bound aluminum; however, aqueous trivalent aluminum is considerably more active chemically and biologically (64). Soluble aluminum is toxic to plants in a variety of ways, including formation of root lesions (65) that may weaken the plant, making it vulnerable to disease, or may kill it outright. Coal fly ash leaching studies reveal that even distilled water can solubilize aluminum, but details of the mechanism have not been disclosed (48, 55). The author posits that aerosolized coal fly ash directly settled in soil or brought down in rainwater is damaging plants both from soluble aluminum toxicity and from pH changes (14).

Exposure to air pollution particulates, not necessarily coal fly ash, in sizes ≤2.5 μm in diameter – often designated PM_2.5_ – is especially detrimental to human health (66). Although the specific mechanisms are not well known, epidemiological studies are beginning to reveal some of the adverse consequences of such exposures. As noted above, exposure to PM_2.5_ has been shown to be associated with increased hospital admissions (32), morbidity and premature mortality (33–35), risk for cardiovascular disease (36) and lung cancer (37), lung inflammation and diabetes (38), risk for stroke (39), Alzheimer’s disease (40, 41), onset of asthma (42), renal function in older men (43), low birth weight (44), and reduced male fertility (45). One may therefore reasonably conclude that aerosolized coal fly ash, at least the PM_2.5_ component, is harmful to human health.

Coal fly ash occurs with grain sizes down to ~0.1 μm in diameter (67). In principle, extracting an ultra-fine fraction of coal fly ash is relatively simple and inexpensive using cyclone classifiers (separators). Certainly, such an ultra-fine fraction would be advantageous for aerial spraying due to added loft time. But there is a serious downside: the toxic elements of coal fly ash tend to be concentrated in the ultra-fine fraction (55). It is not known whether this mechanism for producing ultra-fine enrichment is being used for the covert tropospheric emplacement, but if it is, then that component would be even more toxic than typical coal fly ash.

The toxins in coal fly ash make that substance especially injurious to human health. The small particle size of aerosolized coal fly ash (PM_2.5_) enables particulate intake through inhalation, ingestion, and induction through eyes or skin (68). When inhaled, PM_2.5_ particles can penetrate and become trapped in terminal airways and alveoli, and retained for long periods of time. Here, it can cause inflammation and injury through antagonistic contact (69), through *in situ* toxin release by body moisture (70), and through ionizing radiation from uranium, thorium, and their radioactive daughter products found in coal fly ash (71). Coal fly ash has been described as being more radioactive than nuclear waste (72).

Coal fly ash is able to liberate a host of toxins through exposure to body moisture (70), including aluminum, arsenic, barium, boron, cadmium, chromium, lead, lithium, selenium, strontium, thallium, and thorium and uranium with their radioactive daughter products, and other toxins. Each one of these can have adverse human health consequences, but in combination their synergistic effects may be even more deleterious. Moreover, Haber’s Rule or some more general concentration versus exposure-time relationship may be expected in certain instances where a lower concentration for a long time exposure is approximately equivalent to a higher concentration exposure for a short period of time (16).

The extent of physiological damage from tropospheric coal fly ash is a function of a variety of factors including concentration and exposure duration, as well as the individual’s age, physical condition, and individual susceptibility. Generally, the most at-risk individuals are pregnant women, children, the elderly, and those with compromised immune and respiratory systems. The fetuses of pregnant women exposed to inorganic arsenic from coal fly ash are at risk as arsenic can crossover the placenta. Arsenic can be involved with hypertension-related cardiovascular disease (73), cancer (74), diabetes (75), respiratory diseases (76), and stroke (74). Moreover, arsenic is just one of the numerous toxic elements of coal fly ash that are released by water and by body fluids. Another component, chromium VI, which comprises an estimated 10% of the chromium content of coal fly ash, is not only cytotoxic for lungs and kidneys but is also a carcinogen with the ability to cause lung cancer (77). These examples are just snippets of a vast array of debilitating conditions that can potentially arise from human exposure to aerosolized coal fly ash.

Although aluminum is abundant in Earth’s continental crust, comprising about 8%, it is tightly bound within minerals, and thus is essentially insoluble, i.e., immobile. But coal fly ash is an unnatural product whose aluminum is not so tightly bound. Aluminum in coal fly ash can be extracted in a chemically mobile (soluble) form by water or *in situ* by body fluids (70). Aluminum is implicated in neurological diseases such as Alzheimer’s, autism spectrum disorder (ASD), Parkinson’s, and attention-deficit disorder (ADHD) (49, 51, 78–80), all of which have increased markedly in recent years. Moreover, aluminum is thought to reduce fertility in men (81) and is implicated in neurological disorders of bees and other creatures (82–84).

As might be expected of a covert operation, there have been no public disclosures identifying the principal substance being sprayed, no informed consent, no health warnings, and no serious investigation of the adverse health consequences. The data described here, however, provide strong evidence that the main aerosolized substance being sprayed is coal fly ash; public health inferences can be drawn from extent literature, some of which is cited herein. These citations only provide glimpses of the potential risks involved, but they are sufficient to suggest the possibility of a multi-dimensional global public health crisis, a slow pandemic in the making.

### Potential Unforeseen Hazards Inferred from Fibrous Mesh

From observations, photographic and video evidence, patent literature, and airline pilots’ statements there appears to be two main methods for dispersing the particulate matter in the troposphere: (1) blowing or pumping the powder through nozzles; and (2) dumping large quantities of the powder for the winds to spread. The evidence of a fibrous form of coal fly ash disclosed here presents the possibility of a third dispersing mechanism, one that may pose yet further public health risks.

The author can envision no practical reason for coal fly ash to be deliberately converted into an aerial fibrous form. Moreover, the fibrous form is only sporadically observed, which suggests it is the result of the occasional failure of a specific dispersing mechanism for particulate spray. This fiber-producing mechanism is different in that it involves a heat source, necessary to liquefy the material that generates fibers, a progenitor matrix that may contain additives in addition to coal fly ash, and a motive-mechanism for elongating the liquid into fibers. One known mechanism for producing fibers is to inject a liquid into a blowing stream of air, which causes elongation (85, 86). In principle, fluid drops of coal fly ash and its additives when subjected to the high speed jet combustion exhaust under appropriate physical conditions may be lengthened to form fibers. Two potential processes come to mind that might result in coal fly ash being exposed to jet fuel combustion temperatures: (1) the coal fly ash powder, which may contain dispersion-assisting additives, is injected into the proximity of the jet engine combustion chamber, or (2) the coal fly ash is suspended in the jet fuel, possibly added along with a surfactant at the refinery or fuel distribution center.

The exposure of coal fly ash to the jet fuel combustion environment has further – and perhaps unanticipated – global public health consequences.

As is well known, coal fly ash contains mercury (87–91) in concentrations of 0.1–1.1 μg/g, which may be expected to pollute the environment with mercury as the aerosolized coal fly ash settles to the surface or is brought down by precipitation. Mercury is readily volatile; the possibility should be considered that at elevated temperatures in the presence of copious hydrocarbons, such as are found in the jet fuel combustion environment, conceivably, toxic methylmercury (CH_3_Hg) might form, and be released into the environment. This could explain the methylmercury recently discovered in California fog (92). To the author’s knowledge, this explanation has not been previously considered, and the author could not find either experimental verification or theoretical justification in the scientific literature. Experimental verification should be relatively straightforward. In addition, those who measure methylmercury in fog might look for other toxic gases that might have been produced from coal fly ash at elevated temperatures in the presence of copious hydrocarbons in the jet fuel combustion environment. One possibility that comes to mind is arsine, AsH_3_, but there may be others; this is an unexplored potential area of investigation.

Coal fly ash contains readily volatile chlorine, ca. 200 μ/g (93), and fluorine, ca. 225 μ/g (94). At elevated temperatures in the presence of copious hydrocarbons, such as are found in the jet fuel combustion environment, conceivably chlorine and fluorine might react to form chlorinated-fluorinated hydrocarbons capable of damaging Earth’s ozone layer (95, 96). This could explain the observed post-Montreal Protocol emissions of those ozone-layer-damaging compounds (97). But, as in the case of methylmercury, experimental verification is extremely important because of the potentially profound implications.

### Geophysical Considerations

Within the academic community, there has been some debate as to whether substances emplaced high in the stratosphere will have the intended result of cooling Earth to counteract global warming (18). There is no debate, however, in the open scientific literature on the efficacy of the ongoing covert tropospheric emplacement of aerosolized particulate matter. There should be. Geophysical considerations provide a basis for that discussion.

Although there is no open (unclassified) scientific literature on aerosolized coal fly ash, there are some published articles on the effects of carbon/soot particles. Although coal fly ash may be less efficient than carbon black, generally its effects are similar. Coal fly ash sprayed into the troposphere is expected to inhibit radiation from Earth into space and to heat the atmosphere (98). Coal fly ash particles, settling atop glaciers, will aid in their melting (99).

In copious amounts aerosolized coal fly ash particles, like other pollution particulates, will inhibit rainfall by preventing the smaller water droplets from coalescing and growing large enough to form raindrops (see footnote text 15). Moreover, coal fly ash is hygroscopic. Having formed under anhydrous conditions, it traps water droplets, further inhibiting rainfall. Furthermore, the particulate pollution heats the atmosphere (by absorbed solar energy) and retards heat loss form Earth; consequently, this produces an artificial increase in local atmospheric pressure, which blocks incoming weather fronts, additionally limiting rainfall. Rather than cooling Earth, aerosolized coal fly ash enhances global warming. It also has potentially devastating effects on habitats, including agriculture, from changes in natural weather patterns, from changes in soil pH, and from multiple toxic substances that derive from the coal fly ash.

For at least 15 years, covert weather/climate modification activities have been taking place that involve spraying pollutant particles into the troposphere as observed by many thousands of individuals (see footnote text 2–14). Yet none of the consequences of this near-global weather/climate modification activity has been taken into account by any of the climate change models evaluated by the United Nations’ Intergovernmental Panel on Climate Change (IPCC), which calls into question their validity.

As a weapon aerosolized coal fly ash can be used to cause droughts and concomitant livestock deaths and human starvation. Worse, as discussed above, coal fly ash is a multi-component environmental public health hazard, a slow pandemic that may already be evident in the observed increase in neurological diseases.

## Conclusion

The research results reported here provide strong evidence for the author’s hypothesis: coal fly ash is likely the aerosolized particulate emplaced in the troposphere for geoengineering, weather modification and/or climate alteration purposes. The rainwater element ratios show that the aerial particulate matter has essentially the same water-leach characteristics as coal fly ash. The HEPA air filter dust element ratios occur in the same range of compositions as coal fly ash, as do the element ratios in fibrous mesh found on grass after snow melted.

The documented public health associations for PM_2.5_ particulate pollution are also applicable to aerosolized coal fly ash, which is similar in grain size. These associations include increased hospital admissions, morbidity and premature mortality, low birth weight, lung inflammation and diabetes, risk for cardiovascular disease, lung cancer, lung inflammation and diabetes, risk for stroke, Alzheimer’s disease, onset of asthma, renal function in older men, and reduced male fertility.

The ability of coal fly ash to release aluminum in a chemically mobile form upon exposure to water or body moisture has potentially grave human and environmental consequences over a broad spectrum, including implications for neurological diseases, reduced male fertility, neurological disorders of bees and other creatures, and biota debilitation.

The ability of coal fly ash to release heavy metals and radioactive elements upon exposure to body moisture has potentially grave human health implications over a broad spectrum, including, but not limited to, cancer, cardiovascular disease, diabetes, respiratory diseases, and stroke.

Toxic methylmercury and ozone-damaging chlorinated-fluorinated hydrocarbons, the author posits, may be produced from certain types of tropospheric spraying that places coal fly ash in the jet-fuel combustion environment. Experimental verification is warranted.

From a geophysical perspective, coal fly ash sprayed in the troposphere warms the atmosphere, blocks heat from Earth radiating back into space, and retards rainfall, which can artificially elevate atmospheric pressures that can block incoming weather fronts, further leading to drought conditions. If anything this activity contributes to global warming, the purpose of this covert activity is unknown to the scientific community and to the public. The time has come for the scientific community and especially the environmental science and public health communities to understand that a multiplicity of toxic substances is being sprayed into the air breathed by people in many parts of the world and that it will adversely affect virtually all life on Earth.

## Author Contributions

The author confirms being the sole contributor of this work and approved it for publication.

## Conflict of Interest Statement

The author declares that the research was conducted in the absence of any commercial or financial relationships that could be construed as a potential conflict of interest.

## Footnotes

^1^http://NuclearPlanet.com/AFD-051013-001.pdf

^2^http://globalskywatch.com

^14^http://www.guardacielos.org

^15^http://nuclearplanet.com/NASA_Particulates_Effect_on_Rainfall.pdf

^16^https://www.youtube.com/watch?v=tp2wWuqfbi0

^20^https://www.youtube.com/watch?v=RbwbhzCgGYw

^21^https://www.youtube.com/watch?v=qpysApXRXYE

^24^https://www.youtube.com/watch?v=8KLU2kATAvQ&feature=youtu.be
